This article has been retracted.

# Inhibition of HDAC4 Attenuated JNK/c-Jun-Dependent Neuronal Apoptosis and Early Brain Injury Following Subarachnoid Hemorrhage by Transcriptionally Suppressing MKK7

**DOI:** 10.3389/fncel.2019.00468

**Published:** 2019-10-25

**Authors:** Liqiang Wu, Shulian Zeng, Yali Cao, Ziyan Huang, Sisi Liu, Huaidong Peng, Cheng Zhi, Shanshan Ma, Kunhua Hu, Zhongmin Yuan

**Affiliations:** ^1^Department of Neurosurgery, The Second Affiliated Hospital of Guangzhou Medical University, Guangzhou, China; ^2^Key Laboratory of Neurogenetics and Channelopathies of Guangdong Province, Ministry of Education of China, Institute of Neuroscience of Guangzhou Medical University, Guangzhou, China; ^3^Department of Pharmacy, The Second Affiliated Hospital of Guangzhou Medical University, Guangzhou, China; ^4^Department of Pathology, The Second Affiliated Hospital of Guangzhou Medical University, Guangzhou, China; ^5^Department of Pharmacology, Zhongshan School of Medicine, Sun Yat-sen University, Guangzhou, China; ^6^Guangdong Province Key Laboratory of Brain Function and Disease, Guangzhou, China

**Keywords:** MKK7, JNK, c-Jun, HDAC4, neuronal apoptosis, subarachnoid hemorrhage, early brain injury

## Abstract

The c-Jun N-terminal kinase (JNK)/c-Jun cascade-dependent neuronal apoptosis has been identified as a central element for early brain injury (EBI) following subarachnoid hemorrhage (SAH), but the molecular mechanisms underlying this process are still thoroughly undefined to date. In this study, we found that pan-histone deacetylase (HDAC) inhibition by TSA, SAHA, VPA, and M344 led to a remarkable decrease in the phosphorylation of JNK and c-Jun, concomitant with a significant abrogation of apoptosis caused by potassium deprivation in cultured cerebellar granule neurons (CGNs). Further investigation showed that these effects resulted from HDAC inhibition-induced transcriptional suppression of MKK7, a well-known upstream kinase of JNK. Using small interference RNAs (siRNAs) to silence the respective HDAC members, HDAC4 was screened to be required for MKK7 transcription and JNK/c-Jun activation. LMK235, a specific HDAC4 inhibitor, dose-dependently suppressed MKK7 transcription and JNK/c-Jun activity. Functionally, HDAC4 inhibition *via* knockdown or LMK235 significantly rescued CGN apoptosis induced by potassium deprivation. Moreover, administration of LMK235 remarkably ameliorated the EBI process in SAH rats, associated with an obvious reduction in MKK7 transcription, JNK/c-Jun activity, and neuronal apoptosis. Collectively, the findings provide new insights into the molecular mechanism of neuronal apoptosis regarding HDAC4 in the selective regulation of MKK7 transcription and JNK/c-Jun activity. HDAC4 inhibition could be a potential alternative to prevent MKK7/JNK/c-Jun axis-mediated nervous disorders, including SAH-caused EBI.

## Introduction

Subarachnoid hemorrhage (SAH) is a severe and devastating cerebrovascular disease with high mortality and disability rates greater than 50% (Sekerdag et al., 2018). Recently, early brain injury (EBI), defined as the harmful events that occur within the first 72 h after SAH onset, has been regarded as the primary cause of a poor outcome for patients (Topkoru et al., 2017). Among different pathological causes, the prevalence of neuronal apoptosis after SAH has been confirmed to be an important contributor to the EBI process (Serrone et al., 2015).

The c-Jun N-terminal kinase (JNK; also referred to as the stress-activated protein kinase) cascade is one apoptotic pathway that appears to be particularly important in neurons (Coffey, 2014). JNKs are phosphorylated and activated in neurons in response to various apoptotic stimuli, including oxidative stress (Espinet et al., 2015), DNA damage (Besirli and Johnson, 2003), ischemia–reperfusion (Chen et al., 2018), and the loss of trophic support (Nayak et al., 2016), wherein c-Jun, a well-defined downstream target of JNK, plays an obligatory role in the death process (Yuan et al., 2009; Gupta and Ghosh, 2017). Recently, JNK/c-Jun-dependent neuronal apoptosis has been implicated in EBI after SAH, and the upstream kinases mixed lineage kinase 3 (MLK3)-MKK7 were evidenced to be required for JNK activation (Yin et al., 2016; Okada et al., 2019). Thus, the identification of new ways to target the MLK3-MKK7-JNK-c-Jun cascade would be a promising strategy for the treatment of SAH.

The loss of acetylation homeostasis was found to be closely associated with neuronal apoptosis and nervous system diseases (Saha and Pahan, 2006; Wu Y. et al., 2017). The inhibition of histone deacetylase (HDAC) has been demonstrated independently to prevent neuronal apoptosis induced by oxidative stress or DNA damage. Furthermore, several nervous diseases, including SAH, Alzheimer’s disease (AD), Parkinson’s disease (PD), Huntington’s disease (HD), and ischemia, were ameliorated with obvious decreases in apoptosis after the administration of HDAC inhibitors (Kukucka et al., 2013; Didonna and Opal, 2015; Shao et al., 2016), which suggests that HDACs play crucial roles in the apoptotic neurons suffering from extreme stimuli. However, the related mechanisms remain largely elusive.

In this study, we found that the inactivation of HDACs resulted in a transcriptional suppression of MKK7, concomitant with a reduction in JNK/c-Jun activity and neuronal apoptosis. Further investigation showed that MKK7 transcription critically depended on HDAC4 activity, and the inhibition of HDAC4 effectively suppressed MKK7 expression and JNK/c-Jun-dependent cell death. Moreover, SAH-induced EBI was ameliorated with obvious decreases in MKK7 transcription, JNK/c-Jun activity, and neuronal apoptosis after the administration of the HDAC4 inhibitor LMK235. Our findings highlight that HDAC4 plays a crucial role in sustaining MKK7 transcription and JNK/c-Jun activation in neurons and the inhibition of HDAC4 might be a new strategy to target the cascade for the treatment of SAH.

## Materials and Methods

### Neuronal Culture and Potassium Deprivation

Cerebellar granule neurons (CGNs) were prepared from 7- to 8-day-old Sprague–Dawley rat pups as previously described (Yuan et al., 2009; Wu Y. et al., 2017). Briefly, neurons were dissociated from freshly dissected cerebella and digested into single cells by trypsin in Krebs buffer. Then, 1.0 × 10^6^ cells/ml were seeded in basal medium eagle (BME) that contained 25 mM KCl and 10% fetal bovine serum. Twenty-four hours after seeding, cytosine arabinoside (10 μM) was added.

Potassium deprivation was performed as previously described (Yuan et al., 2009; Wu Y. et al., 2017). Briefly, cells cultured *in vitro* for 7 days (DIV 7) were switched into serum-free BME medium that contained 25 mM KCl (25K) or 5 mM KCl (5K). The HDAC inhibitors SAHA, M344, VPA, and TSA and the HDAC4 inhibitor LMK235 were purchased from Selleck Chemicals (Shanghai, China).

Apoptosis rate was determined by performing nuclear staining with Hoechst 33258 (5 μM) or propidium iodide (or PI, 5 μM) as previously described (Song et al., 2006; Yuan et al., 2009; Wu Y. et al., 2017).

### Western Blotting (WB)

WB analysis was performed to analyze the cell lysis or tissue lysis as previously described in detail (Wu Y. et al., 2017). The supernatants were collected, and the protein concentrations were determined with a BCA kit (Thermo Fisher Scientific, USA). The antibodies used included the following: H3 (CST, #9715), Ac-H3K9 (CST, #9671), Ac-H3K27 (CST, #4353), Caspase 3 (CST, #9662), c-Jun (BD, 610327), p-c-Jun (CST, #9164), MKK7 (EPITMICS, #1949-1), p-SAPK/JNK (CST, #9251), JNK (SCB, #sc-7345), GAPDH (CST, #2118), p-MKK7 (CST, #4171), Tubulin (Sigma, T4026), CST: Cell Signaling Technology (USA), and SCB: Santa Cruz Biotechnology (USA). Horseradish peroxidase-conjugated secondary antibodies were used (Jackson ImmunoRes), and signals were visualized *via* an ECL chemiluminescence system. Representative images from at least three independent experiments are shown, and the relative density analysis for the WB results was analyzed as previously described (Wu Y. et al., 2017).

### Quantitative PCR (Q-PCR)

The TRIzol reagent (Invitrogen) was used to extract total RNA from CGNs or brain tissue as previously described (Wu Y. et al., 2017). Quantitative PCR (Q-PCR) was performed in triplicate on an ABI Prism 7700 sequence detection system using ABI Sybr Green PCR mixture as described by the manufacturer. Actin was used as control and for normalization. Standard procedure for two-step PCR amplification: Stage 1: 95°C 30 s; Stage 2: 95°C 5 s, 60°C 31 s, 40 cycles. Relative RNA expression was calculated using the formula ratio 2^−ΔΔCt^. Data shown represent the mean and S.D. of three separate experiments. The following specific primers were used to amplify *mkk7* (forward, 5′-CAGCGTTATCAGGCAGAA-3′, and reverse, 5′-CAGGATGTTGGAGGGTTT-3′); *actin* (forward, 5′-CAACTGGGACGATATGGAGAAG-3′, and reverse, 5′-TCTCCTTCTGCATCCTGTCAG-3′).

## Immunofluorescence

Immunofluorescence was performed as previously described (Wu Y. et al., 2017). Briefly, the perfusion–fixation or the frozen brain samples were cut into 20-μm sections. One slice was selected from every six serial cuttings in each segment, and four to six slices were collected for immunofluorescence. The slices were subsequently subjected to blocking, primary and secondary antibody incubation, and nucleic staining with Hoechst 33258. Photos were then obtained using a Confocal (ZEISS, LSM 880) or fluorescence-inverted microscope (IX-71, Olympus). The antibodies against MKK7 (EPITMICS, #1949-1), p-c-Jun (CST, #9164), and Cleaved Caspase-3 (CST, #9661) and monoclonal antibody against NeuN (Merck, #MAB377) were used at a dilution of 1:400, 1:400, 1:100, and 1:1,000, respectively.

## RNA Interference

Two HDAC4 small interference RNAs (siRNAs), including siHDAC4-a 5′-GGUCAUGCCAAUCGCAAAUTT-3′ and siHDAC4-b 5′-UUCUGAAGCAUGUGUUUCUTT-3′, and the nonsense control (NC) 5′-UUCUCCGAACGUGUCACGUTT-3′ were used. The interference efficiency of the HDAC4 siRNAs was determined by RNAiMax (Invitrogen) according to the manufacturer’s protocol in rat C6 glioma cells, which were obtained from the Type Culture Collection of the Chinese Academy of Sciences (Shanghai).

DIV5 CGNs were transfected with NC and the siRNAs, together with pEGFP to mark the transfected cells using the calcium phosphate coprecipitation method, and the determination of the interference efficiency of the siRNAs in CGNs has previously been described (Yuan et al., 2009; Kristiansen et al., 2010; Bardai et al., 2012). The apoptotic rate was determined by scoring the percentage of the GFP-positive neuron population with pyknotic nuclei. More than 500 cells for each group were scored blindly without knowledge of their previous treatment.

## SAH Animal Model

Adult female Sprague–Dawley rats (250–280 g, RRID: RGD_70508) were obtained from the Experimental Animal Center of Sun Yat-sen University (Guangzhou, China). The rats were housed at a constant temperature (25 ± 2°C) and air humidity (50 ± 10%), with a 12-h light/dark cycle and free access to water and food. All experimental procedures were conducted under the guidelines of the Institutional Animal Care and Use Committee of Guangzhou Medical University (2015-070). The SAH model was induced *via* the endovascular perforation method as previously described (Wu Y. et al., 2017). For the sample size estimation, the preliminary data showed that there was at least a 10% difference in neuronal apoptosis between the groups, with a standard deviation of 0.07. Therefore, a minimum of six animals per group were required to detect such a difference at 95% confidence (*α* = 0.05) and 0.8 power. The study was not preregistered prior to observing the outcomes or analyzing the data.

## Drug Administration

Drug administration was performed as previously described (Wu Y. et al., 2017). Briefly, the optimum concentration of HDAC4 inhibitor LKM235 (Selleck Chemicals, China) was determined by injecting the inhibitor into the right lateral ventricle of normal mice at 5, 10, 20, and 30 mg/kg, respectively, three mice per dose, and vehicle as a control. LMK235 at 20 mg/kg was chosen for a further test based on the effect of increasing Ac-H3K9 but without affecting behavior and neurological score compared to the control. The LMK235 (20 mg/kg; 100 μl/kg) or vehicle (100 μl/kg) was injected into the right lateral ventricle 24 h prior to SAH induction using the following parameters: 1.5 mm posterior and 1.0 mm right lateral to bregma; 3.7 mm below the horizontal plane of bregma.

## Experimental Designs

### Experimental Design 1

To assess the expression of MKK7, JNK, p-JNK, c-Jun, and p-c-Jun and evaluate the neuronal apoptosis and neurological score, 55 rats were used, including sham: 24 rats and SAH: 31 rats (seven rats died). The animals that died were excluded from further analysis. Both the sham rats and SAH rats were randomly divided into four subgroups according to the required assessments (1, brain water content; 2, IF, TUNEL staining; 3, WB; 4, Extraction of mRNA; *n* = 6 for each subgroup) by running the “RAND” command in Excel software. The clinical scores were recorded prior to anesthesia, and the animals were sacrificed by ventricle perfusion at 24 h post SAH.

### Experimental Design 2

Sixty-seven SAH rats were randomly divided into two groups: the SAH + vehicle group (35 rats, 11 rats died) and the SAH + LMK235 group (32 rats, eight rats died). The two groups were further randomly divided into four subgroups according to the required assessments (1, brain water content; 2, IF, TUNEL staining; 3, WB; 4, extraction of mRNA; *n* = 6 for each subgroup).

Animal experiments were performed based on the timeline diagram shown in Supplementary Data, Supplementary Figure S2.

## Measurement of Brain Water Content

Brain edema was measured using the wet-weight/dry-weight method as previously described (Wu Y. et al., 2017). The brains were removed at 24 h after surgery and separated into the left hemisphere and right hemisphere. The brain samples were subsequently weighed before (wet weight) and after (dry weight) drying in an oven at 105°C for 72 h. The brain water content was calculated as (wet weight − dry weight)/wet weight × 100%.

## Clinical Evaluation

Clinical scores were evaluated by experienced experimenters who were blinded to the experimental grouping as previously described (Wu Y. et al., 2017). Three behavioral activity examinations (Table 1), including appetite, activity, and neurological deficits, were used in the scoring methodology (Zhang et al., 2016).

**Table 1:** Behavior scores.

Category	Behavior	Score
Appetite	Finished meal	0
	Left meal unfinished	1
	Scarcely ate	2
Activity	Walk and reach at least three corners of the cage	0
	Walk with some stimulation	1
	Almost always lying down	2
Deficits	No deficits	0
	Unstable walk	1
	Impossible to walk	2

### TUNEL

TUNEL staining was performed as previously described (Wu Y. et al., 2017). At 24 h after sham or SAH induction, the brains were embedded with paraffin, and the samples were cut into 4-μm sections The index of apoptosis was expressed as the ratio of TUNEL-positive cells to the total number of cells counted in six cortical microscopic fields × 100% in each section (at ×400 magnification). The final average percentage of TUNEL-positive cells of the three sections was used for further analysis of each sample.

### Statistical Analysis

The statistical software SPSS version 18.0 was used for the statistical analysis. Data were determined to be normally distributed prior to analysis. Student’s two-tailed *t*-test was used for comparison between two different groups, and ANOVA was used with Fisher’s LSD multiple-comparison test for multiple comparisons. Data were presented as means ± standard derivations. All *P*-values < 0.05 were considered to be statistically significant, *n* ≥ 3.

## Results

### The Effects of Inhibition of HDACs by pan-HDAC Inhibitors on Neuronal Survival and Apoptosis

To observe the effects of inhibition of HDACs on neuronal survival and apoptosis, cultured CGNs were treated with three types of broad-spectrum HDAC inhibitors (pan-HDAC inhibitors, pan-HDACIs), including hydroxamic acids (TSA and SAHA), synthetic benzamide derivatives (M344), and short-chain fatty acids (VPA). We found that exposure cells to pan-HDACIs for 1 h results in an increase in the levels of H3 lysine 27 and H3 lysine 9 acetylation (Figure 1A), which suggests that the activities of HDACs are efficiently blocked. Prolonging the exposed time of HDACIs to 24 h in 25K media (survival condition) did not induce an increased apoptosis as there were no significant differences in the nuclear pyknosis rates and Caspase 3 activation between the control and the respective HDACI used (Figures 1B,D). In contrast, the administration of the HDACIs remarkably decreased the apoptotic rates evoked by 5K media (apoptotic stimuli) compared with the control (Figure 1C, *P* < 0.05), paralleling with the reduced Caspase 3 activity (Figure 1E). The results suggest that the inhibition of HDACs did not induce obvious cell death, while it prevented neurons from 5K-induced apoptosis.

**Figure 1:** Inhibition of histone deacetylase (HDAC) activity rescued 5K-induced apoptosis. **(A)** DIV 7 cerebellar granule neurons (CGNs) treated with the HDAC inhibitors TSA (500 nM), SAHA (1 μM), M344 (1 μM), or VPA (6 mM) for 1 h were subjected to Western blotting (WB) to detect the levels of Ac-H3K9, Ac-H3K27, and H3. **(B,C)** CGNs treated with these HDAC inhibitors in 25K media for 24 h **(B)** or 5K for 12 h **(C)** were subjected to nucleic staining and apoptotic analysis. Fluorescent photos were obtained using an Olympus IX71 microscope (scale bar = 10 μm). The white arrows indicate the apoptotic cells with nuclear pyknosis. The apoptotic rate was determined by scoring the percentage of cells with nuclear pyknosis in total Hoechst-stained cells. Mean ± SD, *P < 0.05 vs. 25K, ^#^*P* < 0.05 vs. TSA, SAHA, M344, or VPA. **(D)** CGNs were treated with the HDAC inhibitors in 25K media for 24 h and Caspase 3 activity was assessed *via* WB, 5K treatment for 24 h as a control. **(E)** CGNs were treated with the HDAC inhibitors in 5K media for 12 h and the Caspase 3 activity was assessed *via* WB, 25K treatment for 12 h as a control. Tubulin was reprobed to verify equal loadings.

### Inhibition of HDACs Led to a Suppression of MKK7 Transcription and JNK/c-Jun Activity

Evidences from different groups and ours have demonstrated that the activated JNK/c-Jun cascade is critical for 5K-induced CGN apoptosis, and MKK7 is the direct upstream kinase for JNK activation (Watson et al., 1998; Reddy et al., 2013; Wu Y. et al., 2017). Indeed, the time course of analysis indicated that MKK7, JNK, and c-Jun are robustly phosphorylated (activated form) following 5K treatment, starting at 1 h and lasting to 4 h posttreatment (Figure 2A), which suggests that MKK7/JNK/c-Jun signal plays an important role in initiation of apoptosis. Interestingly, we found 5K led to a marked increase in the MKK7 mRNA levels at each time point analyzed, as well as MKK7 protein at 2 h and 4 h post 5K (Figures 2B,C). The data suggested that potassium deprivation caused an acute activation of MKK7 by elevating its phosphorylation and transcription levels.

**Figure 2:** MKK7/ c-Jun N-terminal kinase(JNK)/c-Jun cascade was activated under 5K condition, and inhibition of HDACs transcriptionally suppressed MKK7 expression and lowered 5K-evoked JNK/c-Jun activity. **(A–C)** CGNs in 25K and 5K media for the indicated time course were subjected to WB or reverse transcription (RT)-PCR to detect the levels of phosphorylated-MKK7 (p-MKK7), total MKK7, p-JNK, p-c-Jun (ser73), c-Jun by WB, or *mmk7* mRNA by Quantitative PCR (Q-PCR). GAPDH or *actin* was detected to verify equal loadings. **(B,C)** The gray densities of MKK7 were analyzed after normalization to GAPDH in ImageJ software. Mean ± SD, *P < 0.05 vs. 25K. **(D–F)** CGNs in 25K that contained DMSO or 5K media that contained TSA, SAHA, VPA, or M344 for 12 h were subjected to WB to detect the levels of MKK7, p-JNK, p-c-Jun, or c-Jun by WB or Q-PCR to detect the *mkk7* mRNA level. **(E,F)** The gray densities of MKK7 were analyzed as in **(B,C)**. Mean ± SD, *P < 0.05 vs. 25K, ^#^*P* < 0.05 vs. TSA, SAHA, VPA, or M344, respectively.

It has been reported that MKK7 transcription closely depends on HDAC activity in neuroblastoma cells (He et al., 2016). Consistently, the inhibition of HDAC activity by the pan-HDACIs employed substantially suppressed the MKK7 protein and mRNA levels in 5K-treated neurons and consequently reduced the evoked JNK and c-Jun phosphorylation levels (Figures 2D–F). These results suggested that HDAC activity is also required for MKK7 expression in neurons, and HDAC-dependent MKK7 transcription is most likely a common mechanism.

### Inhibition of HDAC4 Transcriptionally Downregulated MKK7 and Lowered the JNK/c-Jun Activities

To identify the specific HDAC member that is involved in the regulation of MKK7 transcription, the MKK7 mRNA levels were determined following the utility of specific siRNAs to silence the respective member of Class I HDAC (HDAC1, 2, 3, and 8) and Class II HDAC (HDAC4, 5, 6, 7, and 9). Interestingly, we observed that knocking down HDAC4 can remarkably reduce the MKK7 mRNA levels in both the human neuroblastoma cell line SK-N-SH and the glioma cell line U251, while knocking down other members had no such effects (Figure 3A, Supplementary Figure S1). Consistently, in the rat C6 cell line, HDAC4 knockdown also caused a marked reduction of MKK7 mRNA and protein (Figure 3B). Furthermore, HDAC4 knockdown in the transfected neurons led to an obvious decrease in the MKK7 staining rates (Figure 3C). The HDAC4 inhibitor, namely, LMK235, suppressed the MKK7 protein and mRNA levels in a dose-dependent manner in the 25K and 5K conditions and consequently caused a reduction in the JNK/c-Jun activities (Figures 3D–F). The results suggested that HDAC4 activity is required for MKK7 transcription.

**Figure 3:** Inhibition of HDAC4 transcriptionally downregulated MKK7 expression and lowered 5K-evoked JNK/c-Jun activity. **(A)** Human glioma cell line U251 was transfected with siNC or the small interference RNAs (siRNAs) against indicated HDAC members (Supplementary Table S1), and *MKK7* mRNA levels were detected by Q-PCR. Mean ± SD, *P < 0.05 vs. siNC. **(B)** Rat C6 glioma cells were transfected with siNC, siHDAC4-a, or siHDAC4-b, and *mkk7* mRNA or MKK7 protein levels were determined by Q-PCR or WB, respectively. Mean ± SD, *P < 0.05 vs. siNC. **(C)** DIV5 CGNs transfected with siNC, siHDAC4-a, or siHDAC4-b together with pGFP plasmids were subjected to IF for HDAC4 and MKK7 co-staining. Photos were obtained using a confocal microscope (scale bar = 20 μm). GFP was used to mark the transfected cells, and the effect of HDAC4 knockdown on MKK7 expression was determined by scoring the percentage of the GFP-positive neuron population with HDAC4 or MKK7 stained. Mean ± SD, *P < 0.05 vs. siNC, ^#^*P* < 0.05 vs. siNC. **(D–F)** CGNs in 25K or 5K media that contained LMK235 at the indicated doses for 12 h were collected to detect the levels of MKK7, p-JNK, p-c-Jun, c-Jun by WB, or *mkk7* mRNA by Q-PCR. Mean ± SD, *P < 0.05 vs. siNC, ^#^*P* < 0.05 vs. 0.1 μM LMK235.

### Inhibition of HDAC4 Suppressed Neuronal Apoptosis

To examine the effects of HDAC4 inhibition on neuronal apoptosis, the rates of the transfected cells with nuclear pyknosis between the control siNC group and siHDAC4 groups were compared. The knockdown of HDAC4 did not induce an obvious increase in nuclear pyknosis in the 25K-treated neurons compared to the control (Figures 4A,B, *P* > 0.05). In contrast, HDAC4 knockdown remarkably abrogated the apoptotic rates evoked by 5K treatment (Figures 4A,B, *P* < 0.05). Furthermore, the inhibition of HDAC4 by LMK235 dose-dependently prevented 5K-induced apoptosis compared with the control (Figures 4C–F, *P* < 0.05). These results indicated that HDAC4 inhibition induces a substantial suppression of neuronal apoptosis.

**Figure 4:** Inhibition of HDAC4 rescues 5K-induced apoptosis. **(A,B)** CGNs were transfected with siNC, siHDAC4-a, or siHDAC4-b together with pCMV-EGFP. After 48 h, neurons were exposed to 5K media for 12 h and subjected to nucleic staining and apoptotic analysis as in Figure 1. Mean ± SD, *P < 0.05 vs. 25K, ^#^*P* < 0.05 vs. siHDAC4-a or siHDAC4-b. **(C–F)** CGNs in 25K or 5K that contained LMK235 at the indicated doses for 12 h were subjected to apoptotic analysis by nuclear staining with Hoechst 33258 or PI. Mean ± SD, *P < 0.05 vs. 25K, ^#^*P* < 0.05 vs. 5K, ^$^*P* < 0.05 vs. 0.1 μM LMK235, ^∧^*P* < 0.05 vs. 0.5 μM LMK235.

### SAH Results in an Increase in Neuronal Apoptosis, Concomitant With an Activation of JNK/c-Jun

To examine whether JNK/c-Jun activation and neuronal apoptosis occur in the EBI following SAH, the rat SAH model was established by using the endovascular perforation method. Throughout the surgery, none of the sham group rats died, while the mortality in the SAH group was 22.5%. The same part of basal cortical brain tissue was obtained for further biochemical tests (Figure 5A). The animals in the SAH group displayed severe neurobehavioral dysfunction at 24 h post-SAH (Figure 5B, *P* < 0.05). The rate of TUNEL-positive cells in the SAH group was higher than that in the sham group (Figure 5C, *P* < 0.05). The active Caspase 3 was mainly stained in cells co-stained with NeuN in the SAH group but with minimal staining in the sham group (Figure 5D, *P* < 0.05). The results suggest that SAH leads to a typical neuronal apoptosis.

**Figure 5:** Subarachnoid hemorrhage (SAH) results in typical neuronal apoptosis, concomitant with JNK/c-Jun cascade activation. **(A)** Representative pictures of brains are shown after surgery. The same part of basal cortical brain tissue was obtained for tests (circled areas). **(B)** At 24 h post SAH, neurobehavioral performance was assessed. **(C)** TUNEL assay was performed to determine the apoptosis rate at 24 h after SAH (scale bar = 50 μm). Mean ± SD, *P < 0.05 vs. sham. **(D,F)** Active Caspase 3 and p-c-Jun (ser 73) were detected by IF at 24 h post SAH, and the positive rates of all NeuN-stained cells were calculated; scale bar = 20 μm in **(D)** and 50 μm in **(F)**. Mean ± SD, *P < 0.05 vs. sham. **(E)** The levels of p-JNK, JNK, p-c-Jun, and active Caspase 3 were determined by WB at 24 h post SAH. Mean ± SD, *P < 0.05.

The WB results showed that SAH caused a significant elevation in phos-JNK, phos-c-Jun, and cleaved Caspase 3 (Figure 5E, *P* < 0.05). The IF assay indicated that the phosphorylated c-Jun levels remarkably increased in the NeuN-positive neurons in the SAH group compared to the sham group (Figure 5F, *P* < 0.05).

Taken together, the results indicate that SAH caused an obvious increase in neuronal apoptosis at the EBI stage, concomitant with a robust activation of JNK/c-Jun.

### Inhibition of HDAC4 Rescues SAH-Induced JNK/c-Jun Activation and EBI Through Downregulation of MKK7

We subsequently examined whether HDAC4 inhibition could cause a suppression of MKK7 transcription and thereby rescue JNK/c-Jun activation and ameliorate EBI.

There was no obvious difference in the SAH severity among the SAH group, SAH + vehicle group, and SAH + LMK235 group after assessing the blood distributed mainly around the Willis circle, and no significant difference was identified in the neurological score severity between the SAH and SAH + vehicle groups (data not shown). As shown in Figure 6A, the administration of LMK235 caused a marked increase in Ac-H3K9, suggesting that the activity of HDAC4 was efficiently blocked. LMK235 caused an apparent decrease in MKK7 expression, as well as its mRNA levels compared with the vehicle (Figure 6B). Consistent with these changes, SAH-induced JNK and c-Jun phosphorylation was significantly alleviated after LMK235 administration (Figures 6A,C, *P* < 0.05). As a result, the rate of TUNEL-positive neurons in the SAH + LMK235 group markedly decreased compared with those in the SAH + vehicle group (Figure 6D, *P* < 0.05). The administration of LMK235 results in a substantial improvement in the neurological score, as well as brain edema at 24 h following SAH compared to the SAH + vehicle group (Figures 6E,F, *P* < 0.05). Taken together, the inhibition of HDAC4 significantly rescues SAH-induced JNK/c-Jun activation and neuronal apoptosis through the downregulation of MKK7.

**Figure 6:** Administration of LMK235 significantly ameliorated the early brain injury (EBI) process with a reduction in MKK7 transcription, JNK/c-Jun activity, and neuronal apoptosis. **(A,B)** The levels of Ac-H3K9, H3, MKK7, p-JNK, JNK, p-c-Jun, GAPDH, or *mkk7* mRNA were determined by WB or Q-PCR at 24 h post SAH in SAH + vehicle rats or SAH + LMK235 rats. Mean ± SD, *P < 0.05, *n* = 6 per group. **(C)** The p-c-Jun (ser 73) was detected by IF at 24 h post SAH, and the p-c-Jun positive rates of all NeuN-stained cells were calculated in SAH + vehicle rats or SAH + LMK235 rats; scale bar = 50 μm. Mean ± SD, *P < 0.05, *n* = 6 per group. **(D–F)** At 24 h post SAH, the differences in the apoptotic rate, neurobehavioral performance, and brain water content in the left or right hemisphere were compared between SAH + vehicle and SAH + LMK235 groups. Mean ± SD, *P < 0.05, *n* = 6 per group. **(G)** A schematic diagram illustrating the potential mechanisms involved in neuronal apoptosis regulated by HDAC4/MKK7/JNK/c-Jun axis. HDAC4 contributes to MKK7 transcription and expression, which subsequently evokes JNK/c-Jun-dependent neuronal apoptosis and EBI following SAH.

## Discussion

In this study, we found that the inhibition of HDACs by pan-HDAC inhibitors could remarkably suppress MKK7 transcription and subsequently caused a decrease in JNK/c-Jun signals in neurons. Furthermore, we identified that HDAC4 activity is required for MKK7 transcription and JNK/c-Jun activation. The inactivation of HDAC4 by specific siRNAs or the pharmacological inhibitor LMK235 resulted in a decrease in the MKK7 expression and JNK/c-Jun activity, which thereby prevented neuronal apoptosis and significantly ameliorated EBI following SAH. Our *in vitro* and *in vivo* data suggest a tight correlation between the HDAC4 activity and MKK7/JNK/c-Jun cascade-dependent neuronal cell death.

Studies from different groups have highlighted that treatments using various HDAC inhibitors can ameliorate neurodegenerative disorders, as well as acute brain injuries, typically associated with an obvious reduction in neuronal apoptosis (Naftelberg et al., 2017; Thomas and D’Mello, 2018). However, among the identified 18 HDAC members, some members (such as HDAC1, HDAC4, and HDAC6) contribute to neuronal apoptosis, while other members (such as HDAC2) promote neuronal survival. This finding indicates that the anti-apoptotic effects of pan-HDACIs are largely derived from the suppression of an (more) overwhelming death signal(s) in neurons in response to extreme stimuli. If so, it would be interesting to find out the predominant death signal pathway with functions that closely depend on HDAC activity.

In the nervous system, the aberrant activation of JNK/c-Jun pathway has been closely associated with excessive neuron apoptosis, which is considered one of the important pathological causes that contribute to neurodegenerative diseases, including AD, PD, and HD, as well as acute brain injury conditions following stroke, ischemia, or bleeding (Sabapathy, 2012; Kumar et al., 2015; Guo et al., 2018). In this regard, many selective inhibitors that interfere with the JNK cascade have been characterized and are under trials to treat various nervous disorders. Some of these inhibitors display greater protection against neuronal death, and several chemical entities that target the signals, such as XG-102 peptide or the SP600125 derivative CC359, have been independently investigated in Phase 1/2/3 clinical trials for stroke, transient ischemic attack, or AD (LeWitt and Taylor, 2008; Kumar et al., 2015). Thus, the current findings suggest that the JNK cascade is an attractive target for CNS disease.

In the process of EBI following SAH or ischemia, multiple MAPK kinase kinase (MAP3K) members such as TAK1 (TGFβ-activated Kinase 1), MLK3, Activation of apoptosis signal-regulating kinase 1 (ASK1), and DLK dual leucine zipper-bearing kinase (DLK) are activated, which actually contribute to JNK activation and neuronal apoptosis (Hu et al., 2012; Zhang et al., 2015; Yin et al., 2016; Cheon et al., 2018; Zhou et al., 2018). This means that functional compensation among the MAP3Ks may occur when targeting one member for treating EBI. MKK7 has been clarified to be the critical kinase in the transfer of signals from the upstream MAP3Ks to intrinsic JNK/Jun cascades (Whitmarsh et al., 1998; Mooney and Whitmarsh, 2004). However, whether MKK7 is a promising target for preventing JNK/c-Jun cascade-mediated nervous disorders remains elusive.

In this study, we demonstrated the following: (1) MKK7 is rapidly phosphorylated and transcriptionally upregulated following 5K treatment, which results in an acute activation of JNK; (2) inhibition of HDACs suppressed MKK7 transcription and JNK/c-Jun activity in the culture neurons and SAH rats; and (3) inhibition of HDACs rescues neuronal apoptosis *in vitro* and *in vivo*. The presented evidence strongly suggests that the suppression of the MKK7/JNK/c-Jun axis by pan-HDACI accounts for the HDAC inhibition-induced prevention of neuronal apoptosis. HDACI-mediated suppression of MKK7 may represent an alternative for preventing JNK/c-Jun cascade-mediated nervous disorders.

The MKK7 transcription identified here is regulated by HDAC4. As a Class IIa HDAC member, HDAC4 is highly expressed in brain cells and its function is closely linked to its subcellular localization (Fitzsimons, 2015; Mathias et al., 2015). In general, CaMK directly phosphorylates HDAC4, inducing 14–3–3 binding and HDAC4 nuclear export (McKinsey et al., 2000a,b), thereby contributing to neuronal survival (Bolger and Yao, 2005; Chen and Cepko, 2009; Chen et al., 2014; Guo et al., 2015). HDAC4 undergoing nuclear accumulation induces neuronal death by repressing the pro-survival factors MEF2, CREB and PPARγ (peroxisome proliferator-activated receptor γ; Bolger and Yao, 2005; Yang et al., 2011; Li et al., 2012), which have become known as the pathological causes for several disease models, such as PD, stroke, and ataxia telangiectasia (Li et al., 2012; Kassis et al., 2016; Wu Q. et al., 2017). However, although our *in vitro* and *in vivo* data clearly indicated that HDAC4 is required for MKK7 transcription and JNK/c-Jun activation, we did not identify a significant increase in HDAC4 nuclear accumulation in 5K-treated CGNs (at 4 h) or SAH rats (at 24 h) compared to 25K or sham ones, respectively (data not shown), probably because the experimental procedures, such as the time window of detection for them, should be optimized or other unknown reasons. Nevertheless, the identification of specific HDAC modules and downstream substrates for cell types or a specific disease would be of paramount importance in overcoming the nonspecificity of pan-HDAC targeting.

In conclusion, we demonstrated that HDAC is a novel regulatory element important for regulating MKK7 expression, the JNK/c-Jun signal, and neuronal cell death. Furthermore, we identified that the activity of HDAC4 is required for MKK7 transcription, and the HDAC4/MKK7/JNK/c-Jun axis is implicated in neuronal apoptosis and EBI following SAH (Figure 6G). Our data suggest that the inhibition of HDAC4 may present a potential alteration for suppressing the proapoptotic roles of MKK7/JNK/c-Jun signaling in neurons.

## Ethics Statement

All experimental procedures were conducted under the guidelines of the Institutional Animal Care and Use Committee of Guangzhou Medical University (2015-070).

## Author Contributions

ZY, LW, SZ and YC designed the research. LW, SZ, YC, ZH, SL, HP, CZ, SM and KH performed research and analyzed data. ZY supervised the study. ZY, LW, SZ and KH wrote the article.

## Conflict of Interest

The authors declare that the research was conducted in the absence of any commercial or financial relationships that could be construed as a potential conflict of interest.
